# Study on Sustainable Agricultural Structure Optimization Method Based on Multiobjective Optimization Algorithm

**DOI:** 10.1155/2022/5850684

**Published:** 2022-06-13

**Authors:** Dingkang Duan

**Affiliations:** Department of Economics, Belarusian State University, Minsk 220030, Belarus

## Abstract

Agricultural sustainable development is one of the themes of human and nature harmonious coexistence. Adjusting and optimizing agricultural structure are an important direction to improve the level of agricultural sustainable development. In this paper, related research status of the sustainable development of agriculture is analyzed; it shows that there is lack of scientific theories guidance for agricultural sustainable development. In order to optimize sustainable development of agriculture industry structure, the guidance theory of and its optimization are studied. Based on multiobjective optimization theory, several key factors that affect agricultural sustainable development and the main target indexes of agricultural sustainable development are analyzed, the mathematical model of the evaluation of the sustainable development of agriculture is established, and the solution to optimize the multiobjective model is studied. Finally, the agricultural industry sustainable development in a certain area is taken as the research object in this paper; the mathematical model and solving method of agricultural sustainable development evaluation are studied; it provides a guidance to optimize the regional agricultural industrial structure and improve the quality of agricultural sustainable development.

## 1. Introduction

Since the twenty-first century, the Earth ecological environment [1–3] has attracted more and more attention from people. Countries around the world have put forward many measures to improve the ecological environment, such as the greenhouse effect, energy conservation and emissions reduction, pollution control, and green development. Along with the pollution control and the improvement of the management system, raising the level of agricultural pollution becoming one of the main factors affects the quality of regional environment. Agricultural pollutant photo is shown in Figure 1.

Figure 1 shows that agricultural pollution refers to in the process of agricultural production and living in rural areas, without reasonable disposal of pollutants to water, soil, and air; it means the pollution is caused by agricultural products. The number of uncertain, randomness, release is wide and its prevention and treatment are difficult, etc. Main pollution can be divided into two aspects: (1) life waste of rural areas. (2) Rural crop production waste. In the process of agricultural production, it is loss of a reasonable use of pesticides, fertilizers, and agricultural film residue in the farmland and improper disposal of agricultural livestock and poultry dung, fetor produced, as well as unscientific aquaculture water body pollution. In recent years, with the rapid rise of animal husbandry scale cultivation, the livestock excrement pollution caused by agriculture also presents the increasing trend. Many large- and medium-sized livestock and poultry farms lack treatment capacity, and the feces are poured into rivers or stacked at random. After these feces enter the water body or infiltrate into the shallow groundwater, they consume a large amount of oxygen, making other microorganisms in the water unable to survive, resulting in serious “organic pollution”.

According to the survey [4–6], it shows that breeding a cow produces pollution of agricultural products mainly put side by side which is more than the waste water produced by 22 people, while the waste water produced by raising a pig is equivalent to the waste water produced by 7 people.

Relevant research institutions and scholars have conducted extensive and in-depth research on agricultural pollution and its control related research results show that the water quality deterioration and eutrophication are the mainly agricultural pollution; the above phenomenon and agricultural nitrogen and phosphorus loss have a very close connection. The main classification of agricultural pollution is shown in Figure 2.

Figure 2 shows that main classification of agricultural pollution can be divided into farming pollution, agricultural pollution of livestock and poultry breeding pollution, freshwater aquaculture pollution, and pollution of rural life.

In recent years, the level of management and the prevention and control concept about water pollution [7–10] in China's agricultural industry have been improved constantly, dominant means of river basin water pollution control gradually shift from the end of the traditional management to the whole process control, and formed three prevention and control policies of “source control, strengthening management, and ecological restoration.” The pollution total amount control was taken as the root of the river basin water environment protection measures. China's pollution total amount control is based on the pollution discharge outlet of the start of the pollutant concentration control and gradually extended to the point source pollutant total amount control. With the effective control of point source pollution and the rising in the proportion of nonpoint source pollution, the total amount control from single point source pollution total amount control of point source and nonpoint source pollution total amount control transfer together. However, the focus of the total pollution load control is still in the source control, the existing pollution source control measures for all kinds of nonpoint source are mainly about pollution load cuts; how to control agricultural nonpoint source pollution in the deep perspective of industrial structure is an important direction of control pollution source in the future.

Agricultural cleaner production [11–14] can be divided into three links: (1) the use of cleaner production of raw materials. (2) The production process of clean production. (3) The product of cleaner production. In addition, high and stable yield of basic farmland construction, garden ecological economy development, comprehensive utilization of agricultural waste, and agricultural nonpoint source pollution control engineering were used to encourage the development of efficient ecological agriculture and organic agriculture. Such as promoting the applicable mode of ecological agriculture technology, building pollution-free agricultural production, gradually realize agricultural structure rationalization process, technology, ecology, and clean production and product's harmless goal, at the same time, increasing the intensity of ecological agriculture science and technology research, technology, and mode of knowledge innovation, setting up an index system of ecological agriculture, a criteria system, and a certification management system, and mobilizing the enthusiasm of the development of ecological agriculture from local enterprises, farmers, and local government in a larger range.

Relevant experts [15–19] suggest that for controlling pollution from the source, it is important to strengthen the related training in the process of farmers in agricultural production. With promoting the construction of ecological agriculture and the cleaner technology in agriculture production, to control pollution of agricultural chemicals, intensify the construction of ecological agriculture, promoting ecological agriculture practical technology mode, concentrating on the training of prevention and control of agricultural nonpoint source pollution and pollution-free agricultural products in the production knowledge, technology, and legal. In terms of organic pollution, it prevents scale livestock and poultry farms, to strengthen the pollution survey of livestock and poultry farms. Carrying out environmental impact assessment on new large livestock and poultry farms helps to make them as far away from drinking water sources and rivers as possible. By application of advanced technology, the pollution treatment facilities are added, the existing of livestock and poultry farm waste is processed, and comprehensive utilization is done. Anaerobic fermentation of animal manure and commodity organic fertilizer production is promoted. In addition, the intensity of law enforcement should be increased and law enforcement inspection group should carry out the prevention and control of agricultural nonpoint source pollution.

In this paper, the status agricultural industry pollution is analyzed, the method of adjusting and optimizing agricultural industry structure is studied to realize the agricultural industry the purpose of the multiobjective optimization. According to the characteristics of the agriculture industry structure, the agricultural pollution and the goal of optimization of agricultural structure indicators are analyzed and combed. On the basis of the above work, the relationship between the agricultural pollution and the optimal objective index is constructed to improve the agricultural industry sustainable development ability. Application of multiobjective optimization model: agricultural industry in a certain area is taken as the research object, to improve its ability of the agricultural industry sustainable development, the agricultural industrial structure in the region characteristic is analyzed, and on the basis of the multiobjective optimization model studied above, a multiobjective optimization model of sustainable agriculture in the region structure has been established, which is used to solve the multiobjective optimization model, to improve the ability of the agricultural industry sustainable development in the region.

The structure of this paper is as follows: Section 1gives a brief introduction to the agricultural industry structure optimization theory and the development present situation and the existence insufficiency and points out the main research content of this article.  Section 2shows the related works and the target optimization model, and the sustainable development of agriculture industry structure optimization method is analyzed, and the agriculture industry structure optimization model is established.  Section 3 shows the case analysis, industrial structure optimization of a regional sustainable agriculture is taken as a research example, the multiobjective optimization method studied in this paper is adopted to guide the region agricultural industrial structure optimization.  Section 4 gives the combining research results in this paper.

## 2. Related Works

For controlling agricultural pollution at source [20–23], improving the regional water environment quality, improving the ability of the agricultural industry sustainable development, the analysis of the characteristics of spatial distribution characteristics and agricultural pollution industry distribution is needed. Application of the multiobjective programming model: the minimum amount of agricultural pollution load is taken as the goal, which is used to solve the agricultural industrial structure optimization and make adjustment strategy, to realize the agricultural industry development and provide a guidance on the basis of environmental protection. The agricultural industry sustainable development constraint: the optimization problem is a typical multiobjective problem, so the multiobjective planning method is an effective way to solve this problem.

### 2.1. Multiobjective Optimization Model

Since 1800s, related research institutions and scholars [24–27] studied the multiobjective optimization problem and put forward the method to solve the multiobjective problem about weigh calculation and handle the contradiction, and a multiobjective optimization problem in mathematics angle decision method was put forward accordingly.  Figure 3 shows the modeling and solving process of multiobjective optimization problem.

Figure 3 shows that multiobjective optimization model is established to determine the control variable, objective function, and constraint condition. A reasonable optimization algorithm is used to solve multiobjective optimization model and optimize agricultural structure adjustment plans.

Until the mid and late twentieth century, through the accumulation of previous work [28–32], multiobjective programming theory is gradually accepted and applied. Multiobjective programming (MOP) can be mainly divided into the traditional multiobjective programming (TMOP), gray multiobjective programming (GMOP), multiobjective dynamic programming (MODP), etc.

TMOP is an important branch of operational research. Based on linear programming, it is a linear planning method to make up for defects such as single objective function and constraint conditions demanding and a kind of developed scientific management mathematics methods. The model can be divided into the objective function and constraint conditions, two basic parts; they usually exist as contradiction between various objective functions. There is no all-absolute optimal objective function at the same time to achieve the optimal solution and the traditional multiobjective programming model to solve the deviation between actual results and target. The variables are minimized as the starting point of the objective function structure, which is based on the past experience and subjective preference in the process of multiple target balance to obtain relatively satisfactory noninferior solutions. In order to solve the balance problem effectively, traditional multiobjective programming model was efficient due to the simple characteristic; it has been widely used in the field of environment optimization. Due to the characteristics and advantages of the multiobjective programming model, it was studied to reduce the pollution load for the purpose of the agricultural industry structure adjustment, which was taken as a kind of pollution source control method.

GMOP is the combination of gray system theory and multiobjective programming. Due to its characteristic of simple principle and convenient calculation, the result is reliable, the combined model has been used in such aspects as control, forecast, and decision-making application, and showed a clear advantage. System internal information is not complete; there will always be part of the information unknown, and the changes in the system are a complex, uncertain process, namely, gray process. The calculation model consists of events, countermeasures, effect, and targets, four basic elements; the method of gray interval is used to reflect coefficient change situation.

In the environmental system, the environmental factors are both quantitative indicators, and the qualitative indexes and these indexes have uncertainty. Therefore, GMOP model is adopted to solve some environmental optimization usually, especially in the optimal allocation of water resources, land resources, etc. GMOP is used to deal with the randomness, fuzziness, and uncertainty of system problems usually; so, it is taken into the category of uncertainty multiobjective programming by scholars.

MODP is used to analyze and solve the problem of coordination in the process of multistage decision optimization mathematical methods. In the optimal solution for dynamic system, this unique method is not only for a moment to make an effective decision but also in a certain period, continually, to make decisions for many times.

### 2.2. Agricultural Industry Structure Optimization

The agricultural industrial structure optimization is a persistent, complex, evolving process. Since the twenty-first century, the national and regional governments adjust agricultural industry structure optimization policies according to certain requirements. However, most of these policies describe the macro adjustment direction qualitatively. The specific optimization and adjustment plan needs to study and formulate a detailed and quantitative industrial structure adjustment plan after comprehensively evaluating the local conditions, resource allocation, and economic development level. In the study of the problem, it needs to take agriculture as a multivariate compound system, and from the perspective of system science, analysis of agricultural system evolution is done to carry on the overall planning. Output, yield, or environmental benefits are taken as the targets to carry out the research, which is the main direction of the current agricultural industry structure optimization and adjustment of agricultural structure. The method studied in this paper is used to directly reflect the adjustment direction, so as to make the corresponding adjustment policies or measures to adjust and optimize the agricultural industry. Currently, the main research methods are as follows: multiobjective programming, input and output analysis, system dynamics, etc.

According to the introduction of Section 2.1, the MOP is mainly used to study multiobjective function optimization problem within a given range. Agricultural structure adjustment and optimization involve various aspects such as society, economy, ecology, and other aspects; they should be coordinated consideration. If only the pursuit of any one goal is maximized and makes adjustment, it will influence the development of other aspects. The multiobjective programming model to multiple decision variables of the interrelated constraints, effective weighing of the pros and cons of various aspects, can quickly select target adjustment scheme of optimization system, which is a great choice to solve this problem.

Input-output model is one of the important methods for macroeconomic forecasting, which has been widely applied and studied. It is the mathematic method of the balance relationship between each industry. The model in the agricultural industrial structure adjustment applied research usually in agricultural production or production as a production factor, economic investment, fertilizer, pollution emissions, and other factors, such as cultivated land as input factors, and then used a series of mathematical methods to quantify the district agricultural economy and industrial structure adjustment of research and analysis. In order to improve the accuracy of the model, the simulation result has a certain practical significance and reference value, the input-output model combined with multiobjective optimization method, which is the main-stream of the industrial structure optimization method. The combined model is used to study the relationship between the economy and reasonable industrial structure.

MODP is a method of quantitative analysis based on feedback control theory, which can be taken as the long-term and dynamic simulation analysis and research. It is mainly used to solve complex social and economic problems, to deal with nonlinear and time lag problem. The perspective of wholeness and completeness of the interaction between each department and link is emphasized in system dynamics, different control strategy change feedback, and run trend of input system is analyzed, which provides system administrators with a variety of scenarios of decision-making plan and management measures. According to the actual observation to get the information of system, the elements were established through information feedback of interdependence and feasible countermeasures and solutions were put forward; the model has been hailed as a “strategic and policy laboratory.”

## 3. Regional Agricultural Structure Multiobjective Optimization Examples

### 3.1. Introduction of a Regional Agriculture Industry Structure

The researching region is located in a humid subtropical monsoon climate zone, with mild and humid climate, warm spring and cool autumn, hot summer and cold winter, and four distinct seasons. Its river basin is a whole landscape belonging to the low hilly land, and rainfall isoline basic is consistent with the strike of the mountains and is increasing with the topography. There is abundant rainfall in this area, with the most rainfall in summer, the second in spring, the second in autumn, and the least in winter. The annual average rainfall is 1500 mm, and the annual average temperature is 15∼16°C. According to the administrative, division of the region can be divided into six blocks, in order to facilitate as described here; they are named *A*, *B*, *C*, *D*, *E*, *F* administrative region in turn. The region land types are as shown in Table 1.

Table 1 shows that the woodlands region is the largest land use type; it covers an area of 3042.6 km^2^, accounting for a total area of 52% followed by farmland area of 1623.1 km^2^, accounting for a total area of 27.83% town covering an area of 628.7 km^2^, accounting for a total area of 10.83% water area of 421.7 km^2^, accounting for a total area of 7.23% in addition to the above several types of other types of land covering an area of 70.3 km^2^, accounting for a total area of 1.23%.

### 3.2. Agricultural Pollution Load Calculation

The mechanism of agricultural pollution source is complex and fuzzy, with the characteristics of randomness, hysteresis, and hard to monitor. The agricultural pollution load of the quantitative calculation and the comprehensive evaluation is the key and difficult point for environmental pollution prevention and control work. Agricultural pollution load calculation method can be mainly divided into experience statistics and mechanism model method, experience statistics output coefficient method and pollution segmentation method, the rainfall difference method, etc. Methods include SWAT model, AnnAGNPS model, and mechanism model of SWMM model.

In this paper, the characteristics of regional agricultural industrial structure are combined; the output coefficient method is used to calculate the pollution load.

(1) The pollution refers to the rural life sewage in people's daily life into the environment. Usually adopt emission coefficient method to calculate; the formula is shown as follows:
  (1) $$\begin{array}{c} Q_{ri}=U_{cz}\times W_{i}, \end{array}$$
wherein *Q*_*ri*_ is the *i*th total annual emissions of pollutants (kg); *U*_*cz*_ is the population of permanent residents in the rural areas; and *W*_*i*_ is the *i*th *t* kind of pollutant emissions per person. The agricultural pollutants are mainly nitrogen, phosphorus, ammonia nitrogen, etc.
(2) Crop nutrients pollution, planting form of irrigation, and drainage and surface runoff in the region are relatively complex; different block fertilization between the structure and the differences of fertilizing generally use the following formula to calculate crop nutrient pollutant loss situation:
  (2) $$\begin{array}{c} Q_{pj}=W_{zj}\times \frac{U_{zj}}{R_{j}}, \end{array}$$
wherein *Qpj* is the crop nutrient pollutants in for the first *j* a land circulation (kg); *W*_*zj*_ is the *j*th type of land farming land use area (km^2^); *W*_*zj*_ is the crop nutrient pollutants in for the *j*th type a land erosion intensity coefficient (kg/km^2^); and *R*_*j*_ is the first *j*th kind of land use type multiple crop index.
(3) The calculation of livestock and poultry breeding pollution, livestock and poultry breeding pollution generation, and discharge in the region can be calculated as follows:
  (3) $$\begin{array}{c} W_{pf}=\sum_{k=1}^{n}\left(\delta_{k1}\times \alpha_{k1}+\delta_{k2}\times \alpha_{k2}\right)\times N_{k}\times \left(1-\beta_{k}\right), \end{array}$$
wherein *W*_*pf*_ is the total amount of livestock and poultry breeding pollution in the area (kg); *δ*_*k*1_, *δ*_*k*2_ are the first *k*th kinds of livestock and poultry dung individual year and urine production quantity (kg), respectively; *α*_*k*1_, *α*_*k*2_ are the *k*th kinds of livestock and poultry dung and urine from the individual types of contaminants, respectively; *N*_*k*_ is for the *k*th kind of livestock and poultry individuals; and *β*_*k*_ is the *k*th kind of livestock and poultry pollution rate itself.
(4) The area and yield estimation method is used to calculate aquaculture pollution; its calculation formula is
  (4) $$\begin{array}{c} L=A\times S, \end{array}$$
wherein *L* is the total amount of the region in aquaculture pollution (kg); *A* is the discharge coefficient for aquaculture area (kg/km^2^); and *S* is the area of aquaculture (km^2^).

According to the related data provided by the governments in the region, the four different agricultural industry contribution degree of different pollutants before the region agricultural industrial structure optimization and adjustment in the regions have been obtained, as shown in Figure 4.

Figure 4 shows contribution degree of four types of pollutants in the area of different agricultural industry, rural life and planting, livestock and poultry breeding and freshwater aquaculture of CODcr, nitrogen oxides, phosphide, and ammonia nitrogen. It shows that under the current agricultural industry structure, different degree of the agricultural industry contributions of different pollutants are not the same. Rural life of pollutants is the main source of CODcr and ammonia nitrogen.

### 3.3. Agricultural Structure Optimization in a Given Area

As is known to all, there are different development levels of the climatic conditions in different areas; the allocation of resources and economic, agricultural industrial structure are also different. The main factors of the agricultural industry pollution also have different influence degrees. According to the information about the research region introduced above, its climate is appropriate, very suitable for agricultural economic development. In recent years, agricultural pollution in this area is serious; it affects the region agricultural economic health development and becomes the bottleneck of sustainable development in order to control the region agricultural pollution in source, improving sustainable development ability, and building multiobjective optimization model of the agriculture industry structure of the region, by adjusting and optimizing agricultural industry structure to improve the ability of the agricultural industry sustainable development in the region.

The basic form of multiobjective programming model is expressed by mathematical form as follows:

(5) $$\begin{array}{c} \left\{\begin{array}{c} \min\;Z_{k}=\sum_{j=1}^{n}a_{kj}\times x_{j},\;\left(k=1,2,\ldots ,r\right),\\ \text{s.t }\sum_{j=1}^{n}c_{ij}\times x_{j}\geq b_{i},\;\left(i=1,2,\ldots ,m\right)\\ x_{j}\geq 0,\;\left(j=1,2,\ldots ,n\right), \end{array}\right) \end{array}$$

wherein *Z*_*k*_ is the objective function; *X*_*j*_ is the decision variables; *a*_*kj*_ is the objective function coefficient matrix; *c*_*ij*_ is the constraint equation coefficient matrix, and *b*_*i*_ is the constraints to restrict constant vector.

In order to improve the sustainable development ability of agricultural industry in the region, the multiobjective optimization model was constructed on the premise to ensure the security of supply of agricultural products, agricultural pollution, and coordinated development of the agricultural industry. Minimum total agricultural output value maximization: agricultural pollution was taken as the goal, the constraint conditions for the region's agricultural industry development goals, farming scale, output, etc. General requirements are as follows: do not affect the local agricultural economic development level under the premise to a certain extent, to minimize the area pollution total amount.

(1) Establishing objective function: adjusting and optimizing agricultural industry structure, it should meet the demand of economic stability, ensuring supply of local residents, the realization of planting, livestock and poultry breeding, and freshwater aquaculture to minimize the total pollutant emissions.
The objective function can be represented as
  (6) $$\begin{array}{c} \min Z=\sum_{i=1}^{6}\left(\sum_{j=1}^{5}a_{j}A_{ij}+\sum_{k=1}^{4}a_{k}A_{ik}+a_{f}A_{if}\right), \end{array}$$
wherein *Z* is the area pollution total emissions (kg); *A*_*ij*_ is the *j*th kind of planting area in partition of the *i*th region; *A*_*ik*_ is the *i*th division in the *k* of livestock and poultry breeding in the region; *A*_*if*_ is freshwater aquaculture in the *i*th the region partition area; and *a*_*j*_, *a*_*k*_, *a*_*f*_ are the discharge coefficients of all kinds of agricultural pollution sources, respectively.
Different pollution sources of different pollutants have different degree of impact on the environment. For the convenience of expression, the area pollution discharge coefficients of all kinds of unity in the form of matrix description, the specific calculation formula is
  (7) $$\begin{array}{c} a_{xi}=k_{1}\times \varphi_{\text{COD}i}+k_{2}\times \mu_{\text{NT}i}+k_{2}\times \tau_{PTi}, \end{array}$$
wherein *a*_*xi*_ is all kinds of agricultural pollution discharge coefficient; *φ*_COD*i*_, *μ*_NT*i*_, *τ*_PT*i*_ are all kinds of pollution sources of CODcr, nitrogen oxides, a nd the discharge coefficient of phosphide, respectively; and *k*_1_, *k*_2_, *k*_3_ are the environment damages of the above three kinds of pollutants, respectively.
(2) Setting constraints: the development of agricultural industry influenced by multiple factors. Based on the characteristics of local agricultural economy development, the following constraints of adjustment of agricultural industry were identified.

To ensure all kinds of economic crops meet with the demand of the normal supply of planting area, its mathematical expression is

(8) $$\begin{array}{c} \sum_{j=1}^{4}\frac{A_{ij}}{R_{j}}\leq A_{iJ}, \end{array}$$

wherein *A*_*ij*_ is the *i*th partition and the *j*th plant area sown in the region; *R*_*j*_ is the cropping index of all kinds of plants; and *A*_*iJ*_ is the *J*th cultivated land ownership in the *i*th partition.

In order to optimize regional environment and reduce agricultural pollution at the same time, it needs to keep the agricultural economy maintain a certain growth. Namely, agricultural pollution cannot be reduced at the expense of the serious damage to agricultural economic development. Therefore, it should ensure that after the agricultural industrial structure adjustment in economic output, changes should be safe and reasonable, within the scope of the mathematical expression:

(9) $$\begin{array}{c} \sum_{i=1}^{6}\left(\sum_{j=1}^{5}a_{ij}\times A_{ij}+\sum_{k=1}^{4}b_{ik}\times A_{ik}+c_{if}\times A_{if}\right)\geq a_{0}\times V_{0}, \end{array}$$

wherein *a*_0_ is the agricultural GDP adjustment coefficient in the region; *V*_0_ is the regional agricultural industrial structure adjustment in front of the agricultural economy gross domestic product; and *a*_*ij*_, *b*_*ik*_, *c*_*if*_ are the *i*th partitions within all kinds of unit output value of the planting, livestock and poultry breeding, and freshwater aquaculture, respectively.

Regional economic security constraints: in the process of agricultural industrial structure adjustment in the region, it should avoid agricultural economic development planning in this area be impacted in a large level. After determined by way of research, after agricultural industrial structure adjustment, the regional agricultural economy value should not be less than 0.8 before the adjustment. Mathematical expression is

(10) $$\begin{array}{c} \sum_{j=1}^{5}a_{ij}\times A_{ij}+\sum_{k=1}^{4}b_{ik}\times A_{ik}+c_{if}\times A_{if}\geq 0.8\times V_{i}, \end{array}$$

wherein *V*_*i*_ is the agricultural output value of the *i*th partitions in the region before agriculture industry structure adjustment.

Aquaculture production constraints: according to the local agricultural industry development planning, determining the ratio between the output value of livestock and poultry breeding industry, the agriculture output value should be controlled in 20%∼36%, and the ratio between the freshwater aquaculture production and agricultural output value should be controlled in 10%∼25%. They are expressed by the following formulas:

(11) $$\begin{array}{c} 0.2\times a_{0}\times V_{0}\leq \sum_{k=1}^{4}b_{ik}\times A_{ik}\leq 0.36\times a_{0}\times V_{0}, \end{array}$$

(12) $$\begin{array}{c} 0.1\times a_{0}\times V_{0}\leq c_{if}\times A_{if}\leq 0.25\times a_{0}\times V_{0}. \end{array}$$

### 3.4. Region Agricultural Structure Optimization Results and Discussion

According to the multiobjective optimization model of the agriculture industry structure established above, solving the optimization model of the region, the structure adjustment and optimization scheme of agricultural industry can be obtained.  Figure 5 shows the multiobjective optimization process of region agricultural industrial structure adjustment.

Figure 5 shows the region optimization process of multiobjective optimization of agricultural industrial structure adjustment, to improve its sustainable development capacity. According to the multiobjective optimization model of the agricultural industry in the region established in Section 3.3, three optimization schemes are obtained. The three optimization schemes are compared with the current agricultural structure in the region; they are called increase production, production and production agriculture industry adjustment, and optimization scheme in turn. Figures 6 and 7 show the agricultural output values of the three optimization schemes, which are compared with the agricultural industry structure before adjustment.

Figures 6 and 7 show that after agricultural industry optimization in the region, its agricultural industry output value and output value change under three different agricultural industry adjustment schemes. It shows that after was adjusted by optimizing agricultural industry in the region: (1) the output of type production plan down 5% type production scheme of output remains unchanged, while type scheme to increase production output increased 3.2%, respectively. (2) The optimized scheme of three had fallen to the region of livestock and poultry breeding production, suggesting that livestock farming on the environment pollution is most affected, to improve the ability of sustainable development of the local agricultural industry, which should be reasonable control of the scale of the local livestock and poultry breeding industry; (3) the output value of agriculture planting industry in three kinds of schemes is different degrees of ascension, thus the agricultural industry of nutrients to the local environmental pollution degree is less than other industries, in ensuring the local agricultural economic output and reducing the pollution to the environment at the same time, to a certain degree increase of the scale of agriculture planting industry. Figures 8∼10 show the three optimized adjustment schemes of the output type and increase of agricultural production, and their different sources of pollution of CODcr, nitrogen oxides, phosphide, and contribution degree of ammonia nitrogen in the region industry.

Figures 8∼10 show that after the agricultural industry region was adjusted by optimizing, the different pollution sources of industry proportion are different under the optimized adjustment schemes. Each pollutant, the extent of damage to environment sustainability, is endless. In the final selection of the agricultural industry, adjustment and optimization scheme should be considered overall; equal attention to both the local agricultural economic development and environmental protection should be paid.  Figure 11 shows the region was adjusted by agriculture industry structure optimization, the pollutants discharge of six administrative regions.

Figure 11 shows that, (1) under the same agricultural industrial structure, the area pollution emissions are different among different administrative regions, where *D* area is the largest pollution emissions; (2) under different agricultural industry structure, pollutant emissions were different under the same administrative area; (3) the area of agricultural industrial structure adjustment for production: regional emissions are less than several other emissions under the agricultural industrial structure; (4) the area of agricultural industrial structure adjustment is for production, after *A*, *B*, *D*, *E* emissions within the administrative region were greater than other kinds of agricultural structure, but *C*, *F* administrative region of the pollutant emissions is less than before the agricultural industrial structure adjustment; (5) after optimization adjustment agricultural industry in the region, it can improve the local economic benefits or reduce the pollutant emissions to a certain extent; these adjustments to a certain extent can improve the ability of the agricultural industry sustainable development in the region; (6) with the economic growth of agricultural region, it will damage to local environment to a certain extent. So, a reasonable way of agricultural industrial structure adjustment should be chosen according to region agricultural economic development planning.

## 4. Conclusions

In this paper, through the consult-related research status quo of the agricultural industry sustainable development, the method of improving the ability of sustainable development of the agriculture industry has been carried out in-depth study. A multiobjective optimization model of improving the agricultural industry sustainable development ability is set up. In order to verify correctness and feasibility of the multiobjective optimization model studied in this paper, a certain region is taken as research example; the study work about improving the ability of its agricultural industry sustainable development is carried out. The characteristics of regional agricultural industrial structure are analyzed; its multiobjective optimization model is established to improve the ability of its agricultural industry sustainable development. After optimizing the agricultural industrial structure adjustment in the region, three optimal alternatives are obtained. They are named as production type, keep production type, and output production, respectively. Three kinds of agricultural structure adjustment schemes above all can improve the ability of the agricultural industry sustainable development in the region. The finial specific optimization solutions should be chosen by combining with local agriculture economic development in the short-term and long-term planning. Based on the research results in this paper, it can provide theoretical guidance to improve agricultural economic benefits and reduce the pollution of the agricultural industry.

Through the analysis mentioned above, based on the analysis of the characteristics of sustainable development of agricultural industrial structure, the key indicators of sustainable development of the agricultural industry are combined; a multiobjective optimization mathematical model for the agriculture industry structure is built based on the multiobjective optimization theory. The method is applied to optimize agriculture industry structure in a certain area, which proved the validations and effectiveness of the proposed method. Therefore, the multiobjective optimization theory can be applied to guide the sustainable development of agriculture industry structure optimization in the future.

## Figures and Tables

**Figure 1:** Agricultural pollutant photo.

**Figure 2:** The main classification of agricultural pollution.

**Figure 3:** The modeling and solving process of the multiobjective optimization problem.

**Figure 4:** The contribution degree of different industries to four kinds of pollutants before the agricultural industrial structure optimization and adjustment.

**Figure 5:** The agricultural industry structure optimization adjustment optimization process.

**Figure 6:** Agricultural output value changes under the different agricultural industrial structure adjustment.

**Figure 7:** Agricultural output values under the different agricultural industrial structure adjustment.

**Figure 8:** Proportion of all kinds of pollution after agricultural industry structure adjustment about production type.

**Figure 9:** Proportion of all kinds of pollution after agricultural industry structure adjustment about keep production type.

**Figure 10:** Proportion of all kinds of pollution after agricultural industry structure adjustment about output type.

**Figure 11:** Pollution emissions in each agriculture regional under different forms of industrial structure.

**Table 1:** The area of land types.

Classification	Covering area (km^2^)	Proportion (%)
Woodland	3042.6	52
Farmland	1623.1	27.8
Towns and villages	628.7	10.8
Waters	421.7	7.2
Others	70.3	1.2

## Data Availability

The data used to support the findings of this study are available from the corresponding author upon request.
